# Correlations of Pituitary Tumor Transforming Gene Expression with Human Pituitary Adenomas: A Meta-Analysis

**DOI:** 10.1371/journal.pone.0090396

**Published:** 2014-03-04

**Authors:** Jian-Qi Xiao, Xiao-Hai Liu, Bo Hou, Yong Yao, Kan Deng, Min Feng, Bin Xing, Wei Lian, Ren-Zhi Wang, Feng Feng

**Affiliations:** 1 Department of Neurosurgery, Peking Union Medical College Hospital, Chinese Academy of Medical Sciences and Peking Union Medical College, Beijing, P.R. China; 2 Department of Radiology, Peking Union Medical College Hospital, Chinese Academy of Medical Sciences and Peking Union Medical College, Beijing, P.R. China.; Harvard Medical School, United States of America

## Abstract

**Objective:**

Pituitary tumor transforming gene (PTTG) is an important paracrine growth factor involved in early lactotrope transformation and early onset of angiogenesis in pituitary hyperplasia. Emerging evidences have shown that PTTG expression may contribute to the etiology of pituitary adenomas; but individually published studies showed inconclusive results. This meta-analysis aimed to derive a more precise estimation of the correlations of PTTG expression with human pituitary adenomas.

**Methods:**

A range of electronic databases were searched: MEDLINE (1966∼2013), the Cochrane Library Database (Issue 12, 2013), EMBASE (1980∼2013), CINAHL (1982∼2013), Web of Science (1945∼2013) and the Chinese Biomedical Database (CBM) (1982∼2013) without language restrictions. Meta-analysis was performed using the STATA 12.0 software. Crude odds ratio (OR) or standard mean difference (SMD) with its corresponding 95% confidence interval (95%CI) were calculated.

**Results:**

Twenty-four clinical cohort studies were included with a total of 1,464 pituitary adenomas patients. The meta-analysis results revealed that patients with invasive pituitary adenomas had higher positive expression of PTTG than those of non-invasive patients (OR  = 6.68, 95%CI  = 3.72–11.99, *P*<0.001). We also found a significant difference in microvessel density between invasive and non-invasive patients (SMD  = 1.81, 95%CI  = 0.39–3.23, *P* = 0.013). However, there were no significant difference in PTTG expression between functional and non-functional patients with pituitary adenomas (OR  = 1.11, 95%CI  = 0.58–2.10, *P* = 0.753). No publication bias was detected in this meta-analysis (all *P*>0.05).

**Conclusion:**

This present meta-analysis suggests that PTTG expression may be associated with tumor invasiveness and microvessel density of pituitary adenomas, while no correlations with functional status was found.

## Introduction

Pituitary adenomas, abnormal growths in the pituitary gland, represent about 15% of primary intracranial neoplasms and are the second most common type of intracranial tumor by histology in young adults in the 20∼34 years age range [1]. The prevalence of pituitary adenomas is 77.6/100,000 in UK, 80.5/100,000 in Switzerland, 94/100,000 in Belgium, and 75.7/100,000 in Malta [2]. Generally, pituitary adenomas are benign but exhibit invasive or recurrent growth [3]. Like other differentiated neuroendocrine tissues, the pituitary gland displays trophic hormone cell plasticity in response to homeostatic and physiopathological conditions [4]. The pituitary gland responds to complex central and peripheral signals by two mechanisms: (1) trophic hormone secretion is exquisitely controlled to regulate homeostasis;(2) developmental or acquired pituitary signals may elicit plastic pituitary growth responses, consisting of either hypoplasia, hyperplasia, or adenoma formation [5], [6]. Pituitary adenomas arise from monoclonal growth and intrinsic genetic defects which are associated with oncogenes, suppressor genes, and genes charging of differentiation [7]–[10]. Growth factors of hypothalamic or pituitary origin may also act on aberrant cells, contributing to their proliferation [11].

Recently, a large number of studies suggest that expression of pituitary tumor transforming gene (PTTG) plays a key role in the development of pituitary adenomas [12]–[14]. Human PTTG, a protein of 202 amino acids, is a newly discovered biological marker of malignancy grades in several forms of cancer, particularly endocrine malignancies such as pituitary adenomas [15], [16]. PTTG gene was initially isolated from rat pituitary cells [17], is abundantly expressed in endocrine-related tumors, especially pituitary, thyroid, breast, ovarian, and uterine tumors, as well as nonendocrine-related cancers involving the central nervous, pulmonary, and gastrointestinal systems [18]. Previous studies have investigated that PTTG is an important paracrine growth factor involved in early lactotrope transformation and onset of angiogenesis [19]–[21]. Over-expression of PTTG causes in vitro cell transformation, results in vivo tumor formation, and stimulates basic fibroblast growth factor (bFGF) expression and secretion [22], [23]. A number of studies have shown that expression of PTTG may contribute to the development and progression of pituitary adenomas [24]–[26]. However, there is also some evidence showing inconclusive results [27]–[29]. In view of the conflicting results from previous studies, we performed a meta-analysis of all available data to provide a more comprehensive and reliable conclusion on the correlations of PTTG expression with human pituitary adenomas.

## Materials and Methods

### Literature search strategy

A range of electronic databases were searched: MEDLINE (1966∼2013), the Cochrane Library Database (Issue 12, 2013), EMBASE (1980∼2013), CINAHL (1982∼2013), Web of Science (1945∼2013) and the Chinese Biomedical Database (CBM) (1982∼2013) without language restrictions. The following keywords and MeSH terms were used: “pituitary adenoma”, “pituitary adenomas”, “pituitary tumor”, “pituitary macroadenoma”, “PTTG”, “pituitary tumor transforming gene”, “hPTTG”, etc. We also performed a manual search to find other potential articles.

### Selection criteria

The diagnosis of invasive pituitary adenomas must meet the following criteria: (1) pituitary adenomas in grade III∼IV and stage C, D, and E were considered invasive according to Hardy classification; (2) damage to adjacent structures such as the parasellar and cavernous sinus and the hypothalamus could be seen on MRI and CT scans; (3) tumor cell invasion was pathologically confirmed in the sellar bone or adjacent dura mater; (4) sellar bone and dura mater were invaded and damaged, and tumors penetrated sphenoid sinus or invaded parasellar vascular and nervous crossroads. If the study could not meet the inclusion criteria, it would be considered non-invasive pituitary adenomas.

In our meta-analysis, included studies must meet all of the following criteria: (1) the study design must be clinical cohort or case-control study; (2) the study must relate to the roles of PTTG expression in human pituitary adenoma; (3) all patients must conform to the diagnostic criteria of pituitary adenoma; (4) the study must provide sufficient information about PTTG expression and clinical or histopathological characteristics of pituitary adenoma; (5) the invasiveness of pituitary adenomas should be evaluated by imaging characteristics or intraoperative observation. If the study could not meet the inclusion criteria, it was excluded. The most recent or the largest sample size publication was included when the authors published several studies using the same subjects. Any disagreements and inconsistencies were resolved through discussions and subsequent consensus. The supporting PRISMA checklist is available as supporting information; see Checklist S1.

### Data extraction

Using to a standardized form, relevant data were systematically extracted from all included studies by two researchers. The standardized form included the following items: language of publication, publication year of article, the first author's surname, geographical location, design of study, sample size, the source of the subjects, source of samples, detection methods, PTTG expression, etc.

### Quality assessment

We evaluated the methodological quality of the included studies according to the Newcastle-Ottawa Scale (NOS) criteria [29]. The NOS criteria included three aspects: (1) subject selection: 0∼4 scores; (2) comparability of subject: 0∼2 scores; (3) clinical outcome: 0∼3 scores. NOS score ranged from 0 to 9; and a score ≥7 indicates a good quality. The supporting NOS score criteria is available in Supplement S1.

### Statistical analysis

We performed the meta-analysis using the STATA 12.0 software (Stata Corp, College Station, TX, USA). Crude odds ratio (OR) or standard mean difference (SMD) with its corresponding 95% confidence interval (95%CI) were calculated. The *Z* test was used to estimate the statistical significance of ORs. The Cochran's *Q*-statistic and *I^2^* test were used to evaluate potential heterogeneity between studies [30]. If *Q*-test shows a *P*<0.05 or *I^2^* test exhibits >50% which indicates significant heterogeneity, the random-effect model was conducted; otherwise, the fixed-effects model was used. We also performed subgroup and meta-regression analyses to explore potential sources of heterogeneity. Sensitivity analysis was performed by omitting each study in turn to evaluate the influence of single studies on the overall estimate. Funnel plots and Egger's linear regression test were conducted to investigate publication bias [31].

## Results

### Baseline characteristics of included studies

A total of 986 articles relevant to the searched keywords were initially identified. The titles and abstracts of all articles were reviewed and 529 were excluded; full texts and data integrity were then reviewed and another 432 papers were excluded. Finally, 24 clinical cohort studies were included in this meta-analysis [12]–[14], [24]–[27], [32]–[48]. Publication years of the eligible studies ranged from 2003 to 2011. The selection process of eligible studies is shown in Figure 1. The distribution of the number of topic-related literatures in the electronic database for the last decade is shown in Figure 2. A total of 1450 patients with pituitary adenomas were involved in this meta-analysis. Overall, 17 studies were conducted in Asian populations and 7 studies in Caucasian populations. The classical immunohistochemistry method was performed to detect PTTG protein expression in 19 studies, 6 studies used real-time reverse transcription polymerase chain reaction (RT-PCR) method to evaluate PTTG mRNA expressions. We summarized the study characteristics and methodological quality in Table 1–2.

**Figure 1:** Flow chart shows study selection procedure. Twenty cohort studies were included in this meta-analysis.

**Figure 2:** The distribution of the number of topic-related literatures in the electronic database during the last decade.

**Table 1:** Baseline characteristics and methodological quality of included studies focused on the relationships of PTTG expression and invasiveness in pituitary adenomas.

First author [Ref]	Country	Year	Tumor invasiveness		Gender (M/F)	Age (years)	Detection method	NOS score
			Invasion PAs	Non-invasion PAs				
Sun HL [12]	China	2013	29	23	29/23	65.0 (60∼72)	Immunohistochemistry	7
Zhang Y [32]	China	2012	22	41	-	-	Immunohistochemistry	5
Shen YL [33]	China	2012	45	18	27/36	41 (8∼67)	Immunohistochemistry	8
Mo K [26]	China	2011	28	22	23/27	14–68	Immunohistochemistry	7
Wu JS [34]	China	2010	26	22	26/22	46.0±0.5	Immunohistochemistry	7
Zhou J [35]	China	2008	29	20	23/26	-	Immunohistochemistry	6
Wang YS [36]	China	2008	21	27	28/20	36.5±9.7	Immunohistochemistry	7
Li J [25]	China	2008	34	17	28/23	39.0 (17∼68)	Immunohistochemistry	7
He XL [37]	China	2008	15	28	21/27	47.5 (19∼73)	Immunohistochemistry	7
Li AJ [38]	China	2007	26	24	17/33	42.7±11.7	Immunohistochemistry	7
ZY [27]	China	2006	30	25	33/27	39.2 (17∼70)	Immunohistochemistry	7
Hu JF [39]	China	2006	12	28	17/23	45.5 (17∼74)	Immunohistochemistry	7
Li YY [40]	China	2006	30	25	-	-	Immunohistochemistry	6
Wang F [24]	China	2005	38	17	20/35	36.0 (22∼65)	Immunohistochemistry	7
Liu JN [41]	China	2004	20	10	18/12	41.5 (20∼72)	Immunohistochemistry	5

PAs  =  pituitary adenomas; M  =  male; F  =  female; NOS  =  Newcastle-Ottawa Scale.

**Table 2:** Baseline characteristics and methodological quality of included studies focused on the relationships of PTTG expression and functional status in pituitary adenomas.

First author [Ref]	Year	Country	Functional status						Gender (M/F)	Age (years)	Detection method	NOS score
			Non-functional PAs	Functional PAs								
				GH	PRL	ACTH	TSH	LH/FSH				
Sanchez-Tejada L [14]	2013	Spain	33	13					25/21	53.0±15.0	RT-PCR	7
Jia W [13]	2013	China	32	14	6	3	1	14	33/37	45.0±12.8	RT-PCR	8
Salehi F [42]	2010	Canada	14	23	22	10	9	11	-	-	Immunohistochemistry	6
Tena-Suck ML [43]	2008	Mexico	21	24					21/23	43.2±9.4	Immunohistochemistry	7
Minematsu T [44]	2006	Japan	50	29	12	6	3	1	-	-	RT-PCR	6
											Immunohistochemistry	
Filippella M [45]	2006	Italy	6	8	14	6	0	11	20/25	46.4 (19∼79)	Immunohistochemistry	7
McCabe CJ [46]	2003	USA	92	16	5	5	3	0	59/62	-	RT-PCR	6
Hunter JA [47]	2003	UK	18	12	5	5	0	0	-	-	RT-PCR	6
Zhang X [48]	1999	Brazil	30	13	10	1	0	0	22/32	-	RT-PCR	6

PAs  =  pituitary adenomas; M  =  male; F  =  female; NOS  =  Newcastle-Ottawa Scale; RT-PCR  =  real-time reverse transcription polymerase chain reaction.

### Quantitative data synthesis

There 24 cohort studies referred to the relationship of PTTG expression with tumor invasiveness or microvessel density of pituitary adenoma. The random effects model was conducted due to significant heterogeneity existed between studies. The meta-analysis results showed that patients with invasive pituitary adenomas had higher positive expression of PTTG than those of non-invasive patients (OR  = 6.68, 95%CI  = 3.72–11.99, *P*<0.001) (Figure 3). We also found a significant difference in microvessel density between patients with invasive and non-invasive adenomas (SMD  = 1.81, 95%CI  = 0.39–3.23, *P* = 0.013) (Figure 4). Nine cohort studies have reported to the relationship between PTTG expression and functional status of pituitary adenoma. However, there were no significant difference in PTTG expression between functional and non-functional patients with pituitary adenomas (OR  = 1.11, 95%CI  = 0.58–2.10, *P* = 0.753) (Figure 5).

**Figure 3:** Forest plots for the relationship between PTTG expression and tumor invasiveness of pituitary adenomas.

**Figure 4:** Forest plots for the relationship between PTTG expression and microvessel density of pituitary adenomas.

**Figure 5:** Forest plots for the relationship between PTTG expression and functional status of pituitary adenomas.

Sensitivity analysis was performed to assess the influence of each individual study on the pooled OR by omitting each individual studies. The analysis results suggested that no individual studies significantly affected the pooled OR (Figure 6), indicating a statistically robust result. The shapes of the funnel plots did not reveal any evidence of obvious asymmetry (Figure 7). Egger's test also displayed no significant statistical evidence of publication bias under any genetic models (all *P*>0.05), suggesting that no publication bias exists.

**Figure 6:** Sensitivity analysis of the association between PTTG expression and biological characteristics of pituitary adenomas. Results were computed by omitting each study in turn. Meta-analysis random-effects estimates (exponential form) were used. The two ends of the dotted lines represent the 95% CI.

**Figure 7:** Begger's funnel plots of the association between PTTG expression and biological characteristics of pituitary adenomas. Each point represents a separate study for the indicated association. Log [OR], natural logarithm of OR. Horizontal line, mean magnitude of the effect.

## Discussion

Pituitary adenomas arise from epithelial pituitary cells and account for 10∼15% of all intracranial tumors [49]. With the development of molecular biology and cytogenetic techniques, substantial advances in the understanding of pathogenesis and progression of pituitary tumors have been made [50]–[52]. Abundant studies have evaluated the roles of PTTG expression in human pituitary adenomas [46], [50], [53]. PTTG is an oncogene found in pituitary adenomas, and its encoded proteins are involved in a variety of physiological processes, such as gene activation, cell transformation, angiogenesis, apoptosis, DNA repair, genetic stability control, etc [54]. Tfelt-Hansen et al have inferred that PTTG is one of the key factors in the occurrence, proliferation, and invasion of a variety of tumors [55]. Zhang et al concluded that the ubiquitous and prevalent expression of pituitary adenoma PTTG suggests that PTTG plays a role in pituitary tumorigenesis and invasiveness [48]. The important role of PTTG prompted researchers to investigate the relationship between PTTG and biological characteristics of pituitary tumors [53], [56]. Raverot et al have demonstrated that expression of the PTTG gene was related to invasiveness of prolactin (PRL) adenomas [57]. However, many studies have also suggested that the expression of PTTG was not significantly associated with tumor invasiveness in patients with pituitary adenomas [58]. Therefore, the relationships between expression of PTTG and biological characteristics of pituitary adenomas is not entirely certain.

In this present meta-analysis, we evaluated the roles of PTTG expression in human pituitary adenomas. Finally, 24 independent cohort studies were included with a total of 1450 pituitary adenomas patients. Our meta-analysis results suggested that high expression of PTTG was closely associated with enhanced invasiveness of pituitary adenomas, indicating that high expression level of PTTG was related to the invasiveness of pituitary adenomas. We also observed that the microvessel density in invasive patients was significant higher than that of non-invasive patients, suggesting that PTTG expression could be an indicator of tumor proliferative activity and might serve as a potential marker of poor prognosis and tumor recurrence for patients with pituitary adenomas. A study by Filippella et al has suggested the association between PTTG and the recurrence of pituitary adenomas in humans, and set the expression level of PTTG more than 3% as the standard for the confirmation of recurrence [45]. These claims align with our findings in the present meta-analysis. Although the exact function of PTTG in the development and progression of pituitary adenomas is not fully understood yet, a potential explanation might be that high expression of PTTG could cause cell transformation and induce aneuploidy with the abundance or absence of PTTG may lead to the dysregulation of G2/M checkpoint surveillance, leading to abnormal mitosis and chromosomal instability [58]–[60]. Nevertheless, we found no significant difference in PTTG expression between functional and non-functional patients with pituitary adenomas, revealing that PTTG expression may be not the major determinant of functional status of pituitary adenomas [61]. All in all, our findings were consistent with previous studies showing that PTTG expression was associated with biological characteristics of human pituitary adenomas. Our findings might also play important roles in the development of pituitary tumors, suggesting that PTTG expression may be a useful biomarker for pituitary adenomas.

This is the first meta-analysis focusing on the relationships between PTTG expression and biological characteristics of pituitary tumors. Nevertheless, our meta-analysis also had some limitations. Firstly, our results may not provide sufficient statistical power to estimate the roles of PTTG expression in human pituitary adenomas due to relatively small sample size. Secondly, the relationship between PTTG expression and tumor invasiveness and microvessel density of pituitary adenoma were only evaluated among Asian population, while no included studies were conducted among Caucasians, African-Americans and Africans populations, which may severely affect the reliability and applicability of our findings. Thirdly, meta-analysis is a retrospective study that may lead to subject selection bias, which could affect the reliability of our results. Fourthly, our meta-analysis failed to obtain original data from the included studies, which may limit further evaluation of potential roles of PTTG in pituitary adenomas patients. Importantly, the inclusion criteria of cases and controls were not well defined in all included studies, which might also influence our results.

In conclusion, the present meta-analysis indicates that PTTG expression may be associated with tumor invasiveness and microvessel density of pituitary adenomas, while no correlations with functional status. Thus, PTTG may be used as a biomarker for early diagnosis of pituitary adenomas.

## Supporting Information

Checklist S1 **PRISMA Checklist.**
(DOC)

Supplement S1 **The Newcastle-Ottawa Scale for assessing methodological quality.**
(DOC)
